# Migration, Remittances and Nutrition Outcomes of Left-Behind Children: A National-Level Quantitative Assessment of Guatemala

**DOI:** 10.1371/journal.pone.0152089

**Published:** 2016-03-22

**Authors:** Jason Davis, Noli Brazil

**Affiliations:** 1 Carolina Population Center, University of North Carolina, Chapel Hill, North Carolina, United States of America; 2 Spatial Sciences Institute, University of Southern California, Los Angeles, California, United States of America; Old Dominion University, UNITED STATES

## Abstract

Historically, Guatemalans have suffered high rates of poverty and malnutrition while nearly ten percent of their population resides abroad. Many Guatemalan parents use economic migration, mainly international migration to the United States, as a means to improve the human capital prospects of their children. However, as this investigation shows, the timing of migration events in relation to left-behind children’s ages has important, often negative and likely permanent, repercussions on the physical development of their children. To illustrate these dynamics, this investigation uses an instrumental variables framework to disentangle the countervailing effects of Guatemalan fathers’ absences due to migration from concomitant remittances on left-behind children’s growth outcomes. Based on national-level data collected in 2000, the investigation reveals that the international migration of a father in the previous year is correlated with a 22.1% lower length/height-for-age z-score for the average left-behind child aged ≤ 3. In contrast, the receipt of remittance income has no influence on the physical stature of a child, which may indicate that migrant fathers with young children are not able to achieve economic success soon enough during their ventures abroad to fully ameliorate the harmful effects caused by their absences.

## Introduction

Poverty and malnutrition, two diabolical conditions that often go hand in hand, remain rampant throughout much of the developing world. Historically, one of the worst performers in reducing poverty and malnutrition in the Western Hemisphere was Guatemala. In 1989, 55.6% of its population lived in poverty [1], while 62.1% of all Guatemalan children under the age of five were stunted [2]. However, in recent years Guatemala has witnessed significant declines in its poverty rate (26.3% in 2006) [1] and stunting prevalence for children under five (48% in 2009) [2]. Adams [3] argues that economic migration, principally the remittances that were generated, was the single most important factor for reducing poverty and malnutrition in Guatemala in the last decade.

Economic migration and the concomitant remittances can be an integral part of a household’s livelihood strategy for alleviating poverty in places such as Guatemala. To put economic migration and the magnitude of remittance flows to Guatemala into perspective, the International Organization for Migration (IOM) [4, 5] estimates that about 10% of Guatemala’s population lived abroad in the first decade of the 21^st^ century. Mohapatra *et al*. [6] reported a six-fold jump in remittance inflows to Guatemala from 596 million in 2000 to over 4 billion US dollars in 2009—representing 10.8% of Guatemala’s GDP for that year. While Adams [3] did not find that remittances changed overall poverty dynamics in Guatemala in 2000—only 1.6% of poor households were moved out of poverty due to remittances—he did find that remittances contributed to a 12.6% reduction in severe poverty. He explains that remittances received by the “poorest of the poor” households in Guatemala accounted for a disproportionate amount of their overall incomes (60%).

*Prima facie*, one can envision that the flow of remittance income to migrant-sending households would lead to improvements in left-behind children’s well-being. For instance, remittance-receiving households can invest these payments in prenatal and general health care and/or improvements in basic household infrastructure (electricity, clean water and sewage systems). Furthermore, remittances might be used to decrease the risk of malnutrition should a household face a negative income shock such as a meager harvest or severe climatic event. Unfortunately, studies have shown that the disruptive consequences of parental absences, especially in the first few years of migration, can neutralize the positive benefits of remittances to human capital formation. The very act of migration can lead to short-term losses in income, including the need to repay debt incurred to fund a migration trip, and can fracture the nuclear family through infidelity and/or the migrant’s abandonment of his/her family [7] leading to the long-term loss of household income. The temporary or long-term loss of a household breadwinner has contributed to poor children’s health outcomes, including higher rates of infant mortality [8, 9], low birthweight [10] and childhood illnesses [11] in migrant-sending households. This investigation quantifies the overall influence of economic migration—teasing out the beneficial income effects of remittances from the disruptive effects of parental absences—on left-behind children’s physical well-being as measured by the WHO’s length/height-for-age (HAZ) international growth standard [12]. Lower HAZ can be indicative of “stunting” that results from chronic undernourishment and/or infections due to poverty [13, 14]. The long-term consequences of low HAZ cannot be overstated, as it has been linked to several later-life health and social development outcomes, including impaired intellectual development, school achievement, high-risk pregnancies, and decreased economic productivity (15–18).

## Background

One of the first studies examining the health effects of migration and remittances on left-behind family members was conducted by Kanaiaupuni and Donato [8] who found, based on Mexican Migration Project data from five Mexican states, that the short-term absence of the household head was correlated with higher incidences of infant mortality. However, they also noted that higher infant mortality was ameliorated when the household received remittances and/or lived in communities with well-established migration networks. These findings were largely bolstered at the national level in Mexico by Hildebrandt and McKenzie [15] and Hamilton *et al*. [9] who also found positive associations between remittance income and infant survival, especially in rural communities. The former study also found higher birth weights in migrant households and the latter found negative associations between recent out-migration by a family member and infant survival. Further work in rural Mexican households found that the absence of a father was associated with an increased odds of a child being ill and 51–79% higher odds of a child experiencing diarrhea [11].

Another line of inquiry that is more pertinent to this investigation compares children’s growth standards to changes in household migration and remittance receipts. A national-level study using two waves (2002 and 2005) of the Mexican Family Life Survey found a strong detrimental effect of migration, defined to include both parental absence and remittances, on HAZ of children aged 3–6 years [16]. The migration effect translated into an approximately 4.0-centimeter decrease in the height of the average 3-year old child. In Ecuador, inconsistent findings based on 2006 Living Standards Measurement Survey data on the effects of remittances on child undernutrition were recently published. Ponce *et al*. [17] found no significant difference in HAZ and weight-for-age z-scores (WAZ) for children aged <5 living in households receiving remittances. In contrast, Antón [18] identified a statistically positive association between remittances received and z-scores for both height for weight (HWZ) and WAZ, while not finding a significant difference in HAZ. Specifically, children aged <5 living in households that received the average amount of remittances for the studied population had HWZ and WAZ values that were 0.74 and 0.06 standard deviations higher, respectively, than non-remittance receiving households. The major difference between the two studies rests with the selection of remittance instrumental variables (IVs): Ponce *et al*. (2011) used exogenous variation in transaction costs for international transfers whereas Anton (2010) used a combination of the number of Western Union offices per capita and the proportion of households with migrants by province.

Studies of economic migration and child development conducted in other geographical contexts have also yielded mixed findings. For example, de Brauw and Mu [19] largely found no association between the internal migration of parents and other family members and the over- and underweight prevalence of children in China. In contrast, Gao *et al*. found significant negative associations between parental migration and unhealthy behaviors amongst left-behind adolescent school children in rural China [20]. Additional work in the Philippines and Vietnam found that economic migration failed to help move left-behind children aged 9 to 11 from a stunted to a non-stunted condition [21]. The non-significant finding may be a function of the fact that stunting is largely set by the third year of life [22, 23].

The closest investigation to the present study was conducted by Carletto *et al*. [24] using primary data collected from the Western Highlands of Guatemala in 2008. They found that HAZ was approximately one half a standard deviation higher and the probability of stunting 6% lower for children aged 0–6 from migrant-sending households compared to demographically similar children from non-migrant households. The present investigation differs from Carletto *et al*. [24] in three substantial ways: (1) Carletto *et al*. lumped remittances within the overall migration effect, whereas this study disentangles the income effects of remittances from the disruptive effects of parental absences due to migration; (2) Carletto *et al*. used a difference-in-differences approach, whereas this study uses IVs to address the endogeneity of decisions to migrate and/or send remittances and children’s health status; and (3) this study uses national-level instead of regional-level data to investigate stunting conditions in left-behind children from Guatemalan migrant-sending households.

## Research Question and Theory

The current study sets out to answer the following research question: How do income remittances and fathers’ migration influence child well-being in migrant-sending households? Specifically, how does the migration/remittance phenomenon influence growth rates in “left-behind” children in Guatemala? We hypothesize that HAZ will be negatively affected by a father’s migration but positively affected by a rise in remittances received by the household. Corresponding theories that bolster the research hypotheses, separating the disruptive effects associated with fathers’ absences from the income effects of remittances, are described below.

### Income Effects

Whether through altruistic motives or enlightened self-interest, migrants who seek wage labor abroad do so with the intention of elevating overall household income [25–27]. As argued by Becker and others, when household income rises (e.g., remittances from international destinations), couples tend to have fewer children but invest more in their children’s human capital through education and health expenditures [15, 28, 29]. Therefore, as household income attributable to remittances rises, investments in children’s health are likely to increase with concomitant reductions in neonatal and infant mortality, illnesses, low birth weight, and underweight young children [15]. Ethnographic fieldwork performed in Guatemala’s Western Highlands provides evidence for this. In response to the question, “How do migrants from your community use remittances?,” over 50% of informants mentioned new home construction, investing in the human capital (education and health) of their children and to cover basic household expenses including food, clothes, fuel, power, water and medicine [30]. Furthermore, all informants couched their responses by stating that these remittance investments, including the building of a new house, were meant to benefit the future prospects of their children. Additional examples in Mexico and Ecuador show correlations among remittances increases, a rise in health expenditures and declines in the prevalence of undernutrition and infant mortality [9, 18].

### Disruptive Effects

The migration disruption hypothesis argues that during the act of migration and the intervening time required to settle in a new location, the normal functioning of the household is disrupted [31, 32]. There are numerous obstacles that migrants face toward achieving their ultimate goal of securing gainful employment and remitting earned income to their families. These obstacles include obtaining sufficient capital to make the migration journey, which may entail obtaining a loan from family or friends, with the loan amount increasing when a *coyote* (human smuggler) is hired to facilitate the migration event. For undocumented migrants, international borders must be successfully crossed before the search for stable and secure employment can begin. Overcoming these obstacles takes time and thus households may be saddled with significant debt that may take years to pay off [33, 34]. These factors may delay the positive income effects outlined in the previous section, which have serious consequences for young children if the delay coincides with their critical period of physical development.

A more holistic view of the migration disruption hypothesis also considers the effects on left-behind household members. In the absence of migrant breadwinners and the immediate receipt of remittance income, left-behind caregivers and dependents must cope until meaningful remittances can be sent [8]. Subsistence strategies for left-behind mother caregivers may include taking on wage labor or farm maintenance activities to compensate for a temporary decline in income attributable to the absence of a breadwinner. When a left-behind mother utilizes these subsistence strategies to compensate for lost labor, her infant child(ren) may be harmed due to a reduction in breastfeeding [35–40] or lack of supervision leading to higher incidences of child illness [11]. Additional research finds that the disruptive effects of economic migration can contribute to higher infant mortality rates [8, 9], increased disease prevalence [11] and slower growth rates [16] in left-behind children.

## Data

To answer the study’s research questions, nationally representative, cross-sectional data from Guatemala’s 2000 *Encuesta Nacional de Condiciones de Vida* (ENCOVI) are used. Guatemala’s ENCOVI provides a rich source of individual, household and municipal-level data that cover 7,276 households (3,852 rural) and over 37,000 individuals. These data were obtained from the World Bank with participant information anonymized and de-identified prior to analysis. The cross-sectional data were collected using a stratified probabilistic sampling design to capture a proportional number of households from each of Guatemala’s 22 departments. In the analysis, we exclude single-parent households due to separation, divorce and the death of a spouse, leaving us with an analytic sample of 3,973 children ≤ 3 years old. There are 244 children who live in households with a missing parent. These parents are likely migrants that are not living in the household during the time of the survey. We imputed their migrant status based on the spouse’s reported location of remittances: 103 received domestic remittances, 78 received international remittances, and 63 received no remittances. Missing parents in the first group are designated as domestic migrants, the second group as international migrants, and the last group are excluded from the analysis. However, including the 63 children from the non-remittances group by designating their missing parents as either all domestic or all international does not alter the results.

We tested the relationship of HAZ with changes in fathers’ international migration status and household remittance receipts during the prior 12-month period. WHO Macro Packages for Stata were used to calculate HAZ [41, 42]. Statistical analyses were performed with children aged ≤ 3 to address the fact that stunting, defined as being < -2 standard deviations of HAZ from the global average [12, 43], is unlikely to occur after a child has reached the age of three [23, 44]. We examined the effects of economic migration on HAZ growth to determine if parental goals for improving children health are undermined by migration timing in relation to a left-behind child’s development status. We also analyzed other WHO international growth standards including WAZ as an indicator of underweight, HWZ as an indicator of wasting and body mass index as an indicator of overweight. Results from these analyses are not included due to their non-significant outcomes.

The key independent variables of interest are fathers’ international migration and the receipt of household international remittances. The father migration variable indicates (1 = yes, 0 = no) whether a child's father has lived internationally at any point in the past year. We exclude from the analysis children of mothers who migrated internationally either by themselves or with their spouses since these cases make up less than 1% of the sample. Our remittances variable indicates (1 = yes, 0 = no) whether a child's household received international remittances in the past year. Since the survey data contain no information on the characteristics of the remittance sender, households may be receiving remittances from members other than a parent.

In the analysis, we accounted for several child- (age, age^2, ethnicity and gender), household- (wealth, size and whether it is rural or urban), and parent-specific (education, age and height) variables. Gender, ethnicity and urbanicity were included because national-level surveys show girls, ethnic Mayan children (compared with ladino) and children residing in rural communities face substantial poverty and discrimination-related barriers to education and health [45, 46]. We included a quadratic term for age since undernutrition expresses itself in a non-linear fashion for young children. Additionally, the number of individuals living in the household is incorporated into the analysis based on research showing a linkage between decreased child quality and larger families [47]. The parent-specific variables controlled for relative differences due to parent’s age and education (older and more educated parents may be better able to feed their children). Through the parent-specific variables, we also controlled for genetic predisposition to shorter stature with father’s and mother’s height. Lastly, we controlled for regional differences by grouping children into the following three categories: 1) Metropolitan, 2) Southwest and Northwest and 3) North, Northeastern, Southeastern, Central and Petén—the largest and northernmost department in Guatemala.

The household asset index is a measure that controls for the relative wealth of the household prior to the year 2000—the year of the survey. Instead of income, which can be highly variable, household assets and infrastructure can provide a better measure of relative wealth, which can influence both migration decision-making and the ability of parents to adequately feed their children. Following the methodology described in Filmer and Pritchett [48] and McKenzie [49], principal components analysis was used to create a household asset index. Father's age (4% of children) and height (16%), and mother's age (< 1%) and height (4%) had missing data, which were imputed using the predicted values from regressing these variables on the rest of the independent variables. Including a set of dummy variables indicating imputed values did not significantly change the results.

## Methodology

In order to estimate the effects of fathers’ international migration and household remittances on child well-being, we estimated the following general relationship:

Y=g(β;X,M,R)+ε, (1)

where *Y* is a continuous measure of HAZ, *X* is a matrix of child and parental control variables, *M* measures the international migration status of the parents, *R* indicates the household receipt of international remittances, *g*(∙) is the response function, and *ε* is an idiosyncratic shock.

We can estimate Eq 1 with a basic linear regression, but the estimated effects are likely biased due to several methodological problems. First, selection is a concern if the characteristics of fathers who migrate and households that receive remittances are also correlated with child well-being [15, 50]. This is likely the case since the estimated effects may be partly driven by unobservable variables, such as parental concern over a child's welfare, that happen to be correlated with a father’s migration status and the receipt of international remittances. Second, economic migration and child well-being may be simultaneously determined, as it is likely that child well-being affects a father’s and household’s economic migration behavior and vice versa [51]. Third, Eq 1 treats children as independent units, but a migrating father and the receipt of remittances similarly affect children living in the same household. It may be unrealistic to assume that the nutrition status of children living in the same household are independent given the observed covariates, or in other words that the child- and household-specific residuals are independent. Lastly, father's migration and household remittances may be subject to the same exogenous shocks, which could result in contemporaneous correlation across the estimated equations.

In order to minimize these methodological issues, we estimated Eq 1 as a system of simultaneous mixed process equations using limited information maximum likelihood [52]. Formally, we estimated the following system of equations:

$$P(M=1|X,MN)=\Phi \left(\beta_{o}+\beta_{1}MN+\beta_{2}X\right),$$ (2)

$$P(R=1|X,WAGE)=\Phi \left(\beta_{o}+\beta_{1}WAGE+\beta_{2}X\right),$$ (3)

$$Y=\beta_{o}+\beta_{1}\hat{M}+\beta_{2}\hat{R}+\beta_{3}X,$$ (4)

Eq 2 models the probability that a father migrated internationally using a probit specification, where Φ is the standard normal cumulative distribution function. Eq 3 estimates the probability a child's household received international remittances. Using a linear specification, Eq 4 estimates our HAZ growth measure as a function of $\hat{M}$, the predicted probability of international fathers’ migration from Eq 2, $\hat{R}$, the predicted probability of receiving international remittances from Eq 3 and a rich set of covariates *X*. Solving Eqs 2–4 simultaneously rather than in stages as single-level equations allows for correlated errors across equations, which controls for contemporaneous correlation across equations and endogeneity due to simultaneity. In order to account for the correlation of nutrition status between children within households, we clustered standard errors at the household level.

To statistically control for unobserved selection into migration and remittance receipts, we postulate that migration and remittances are a function of IVs. We instrumented migration using migration networks *MN*. Previous literature has shown that migration networks significantly influence migration behavior [53–55]. Members of a community who have previously migrated lower the costs of out-migration by sharing information about travel, process and jobs in other areas. Additionally, the more migrants in a community signal a higher success rate, further motivating those who have not migrated to consider leaving their communities to seek opportunities elsewhere. We operationalized migration networks as the percent of households in the municipality that have an international migrant in the past year. The migration prevalence instrument was derived from the 2002 Guatemala Census. The census asked whether anyone from the household migrated internationally in the preceding ten years. We used responses to this question to categorize migrant-sending households as those with at least one member venturing abroad in the preceding decade. Finally, the proportion of migrant versus non-migrant households was extrapolated to the municipality level.

Since the rate of international migration in the past ten years is likely correlated with events in 2000, the year of the survey, and thus correlated with health outcomes measured in 2000, we interacted the variable with unexpected rainfall shocks in 1991. Rainfall shocks have been used in prior research as instruments for migration [56–58]. Drawing from these studies, we argue that because rain is correlated with agricultural production and income, an unexpected drop in rain levels in one year may cause people to migrate, particularly out of rural areas. Unexpected rainfall shocks should be a valid instrument as it is likely to have an important effect in a country such as Guatemala where a majority of households directly or indirectly depend on agriculture as a source of income. We obtained annual municipal level rainfall data (in millimeters) for the years 1990 to 2010 from Guatemala’s *Instituto Nacional de Sismología*, *Vulcanología*, *Meteorología e Hidrología* [59]. In order to account for missing rainfall data, we spatially interpolated the annual rainfall using inverse distance weighting, an interpolation method that averages the rainfall of nearby municipalities, giving greater weight to the closest municipalities. From this yearly data, we estimated a model that predicts the change in rainfall from time *t*-1 to *t* from the level of rainfall in time *t*-1. We then used the residuals in 1991 from this model as the unexpected municipal-level rainfall shock. We measured rainfall shocks in 1991 for the following two reasons. First, we wanted to obtain rainfall shocks in the earliest year possible with the most complete rainfall data. Rainfall data prior to 1991 are significantly incomplete for most municipalities. Second, based on statistical tests unexpected rainfall shocks from 1991 obtained the lowest indicator of potential bias [57].

Although rainfall shocks may be temporally random, they may occur in certain areas (e.g., wet regions) vs. others (e.g., dry regions). This spatial association potentially introduces a correlation between rainfall shocks and unobserved components in the HAZ equation. In order to minimize this potential endogeneity, we controlled for rainfall levels in 1999 in all estimating equations [57].

We instrumented international remittances using the cost of living adjusted average wage rate for non-skilled workers in US migration destinations (*WAGE*). The logic for using *WAGE* as an instrument is that a non-skilled migrant is more likely to remit excess income from areas where the average non-skilled wage rate is higher, *ceteris paribus*. Furthermore, this US non-skilled wage IV only influences children’s health outcomes through its influence on remittance volume to the household. The *WAGE* IV was created in multiple steps following similar methodology described in Adams and Cuecuecha [57]. We first obtained from the International Office of Migration [60] the total remittance transfer estimates in 2004 for each of Guatemala’s 22 departments disaggregated by the 25 US cities (represented by metro area) with the highest remittance income sent to Guatemala. We then converted remittance volume estimates into percentages by US city of origin. Next, we obtained 1998 average non-skilled hourly wage rates for the 25 US cities from the Bureau of Labor Statistics [61] adjusted for differences in cost of living. Finally, we created a weighted-average hourly wage rate at the Guatemalan department level based on the percentage of remittance volume from each US city of remittance origin to that department. To obtain variation at the household level, we interacted this variable with the square of the age of the head of the household.

The validity of our instruments is based on the assumption that migration networks and US destination wage rates affect a father's decision to migrate and each household's remittance level but have no independent effects on child nutrition status. A violation of this assumption occurs if remittances are used to improve community infrastructure that may indirectly improve the growth outcomes of all children in the community. Much of the early work on migrants' remittances suggests that transfers are sent primarily to help meet household needs. However, recent evidence revealed that remittances may finance investments in the community of origin in the form of financial assets and microenterprises [62]. Osili found that remittances sent to finance investments in the origin community are positively associated with origin household resources [63]. Another concern is that migrant-sending communities are more likely to possess greater social capital and collective efficacy, which may help offset the negative impact of a migrating father's absence on his child's well-being. Given these potential threats to the validity of our IVs, we added controls for health care access/exclusion and community cohesion in all equations. Both variables were derived from Guatemala’s 2000 ENCOVI community questionnaire. The health care exclusion variable is a measure of the percentage of community members that do not have access to health care services. This variable controls for differential health infrastructure at the community level that might be influenced by remittance flows. The community cohesion variable is a measure of whether community members are very, somewhat or not willing to loan money to other community members. This variable seeks to control for the fact that residents in communities with stronger migration histories/networks might be more prone to help one another, especially left-behind family members during the more stressful initial years of migration.

We jointly estimate Eqs 2–4 using the Stata 12.0 command *cmp* developed by Roodman [52]. The command generates conditional mixed-process estimators using limited-information maximum likelihood. We used the Likelihood Ratio statistic proposed by Buis [64] to test for the joint significance of our instruments. The test determines whether our instruments jointly suffer from the weak instrument problem [50].

## Results

### Descriptive Results

Mean values of the variables used in the analysis disaggregated by the four migration and remittance categories are presented in Table 1. Approximately 4% of sampled Guatemalan children age 3 and under had a father residing abroad in 2000 and 6% of children lived in households that received international remittances. Of note is the overall poor level of child nutrition in Guatemala. The average child in the sample has a HAZ of -1.931, a value just slightly above stunting status (HAZ ≤ -2). Given such a poor baseline level of nutrition, the migration of a father or an additional stream of income in the form of international remittances may trigger a significant reversal in the health trajectory of a child.

**Table 1:** Mean characteristics of children age ≤ 3 by father's migration status and household remittances receipt in Guatemala^a^.

Variable	Non-migrant, non-remittance-receiving	Non-migrant, remittance receiving	Migrant, non- remittance receiving	Migrant, remittance-receiving	Total
Length/Height-for-Age Z-score (HAZ)	-1.929	-1.569	-2.678	-2.011	-1.931
Child-Specific					
Age	1.464	1.479	1.432	1.577	1.467
Age^2	3.414	3.411	3.432	3.845	3.425
Female	0.486	0.548	0.446	0.526	0.488
Parent-Specific					
Either Parent Mayan	0.499	0.651	0.351	0.433	0.500
Father’s Age	32.248	32.718	31.743	31.945	32.249
Father’s Height (meters)	159.479	161.531	153.909	158.824	159.434
Mother’s Age	28.086	28.295	27.730	25.526	28.025
Mother’s Height (meters)	147.166	150.438	145.478	147.654	147.267
*Parents’ Highest Education Level*					
Below Primary	0.193	0.116	0.378	0.258	0.195
Primary	0.587	0.493	0.486	0.536	0.580
Secondary	0.220	0.390	0.135	0.206	0.224
Household-Specific					
Household Size	6.527	7.952	7.041	6.381	6.585
Household Asset Index	1.583	2.600	1.280	1.805	1.620
Lives in Rural Region	0.653	0.562	0.905	0.660	0.654
Municipal-level					
Rainfall in 1999	1816.017	1804.932	1609.306	1731.802	1809.703
Community Cohesion	2.306	2.205	2.284	2.196	2.299
Health Care Exclusion	21.554	17.370	14.595	13.351	21.070
*Region*					
Metropolitan	0.077	0.137	0.081	0.041	0.078
Southwest and Northwest	0.596	0.370	0.027	0.268	0.569
Other	0.327	0.493	0.892	0.691	0.353
Instrumental Variables					
Community Migration Network^b^	-3.674	-6.066	-70.426	-20.775	-5.423
US Destination Wage Rate^c^	8,517.352	12,835.580	9,766.167	9,450.906	8,722.091
Number of Children	3,656	146	74	97	3,973

Source: 2000 Encuesta Nacional de Condiciones de Vida, Guatemala.

^a^A migrant household means a child’s father or mother has migrated internationally in 2000 whereas a remittance-receiving household means the household has received international remittances from any member of the household in 2000.

^b^ International migration rate in 2002 times unexpected rainfall in municipality.

^c^ Non-skilled wages in the United States in 1998 times the square of the age of household head.

Among the four categories, children living in households with a migrant father that do not receive remittances have the smallest average HAZ (-2.678), indicating a greater degree of stunting. In contrast, children living in remittance-receiving households without a migrant father have the largest average HAZ (-1.569). Furthermore, children whose households do not receive remittances and whose fathers do not migrate (-1.929) and children whose households receive remittances and whose fathers migrate (-2.011) have similar HAZ values. These results suggest that migration has a negative (amplifying) effect and remittances have a counterbalancing positive (dampening) effect on stunting. These initial findings are merely suggestive since they do not account for the observed and unobserved characteristics that may be driving the patterns shown in the table.

### IV Results

Results in Tables 2 and 3 represent our IV model findings. Table 2 presents results from the probit models predicting fathers’ migration status and remittance receipt. The results suggest that mother's age, a parent with a primary education relative to a below primary education and health care exclusion are negatively associated with the probability of a migrating father. In contrast, household wealth and living in areas other than the Metropolitan, Southwest and Northwest regions are associated with higher probabilities of a father migrating internationally. For the probability of receiving international remittances, only mother's age has a negative association. In contrast, children who are female, have older fathers and taller mothers, live in households that are larger and wealthier, and live in areas other than the Metropolitan, Southwest and Northwest regions have a greater probability of residing in households receiving international remittances. The most important result in the table relates to the validity of the instruments. Both instruments show the expected signs and are statistically significant. The negative sign on the father migration instrument indicates that if there is more rainfall than expected, there are fewer international father migrants. The positive sign on the remittances instrument indicates that higher wages for non-skilled labor in traditional Guatemalan remittance sending cities in the US increase the probability of receiving international remittances. The variables also jointly appear to be strong IVs: the Wald Chi-square statistic for the test of the joint significance of the instruments is 79.33, with a p-value significantly less than 0.05.

**Table 2:** Independent and instrumental variable effects on international father's migration and remittance transmission to Guatemala households (N = 3,973).

	Father migrated internationally		Household received international remittances	
	Estimate	(SE^1^)	Estimate	(SE^1^)
Individual controls				
Age	-0.087	(0.114)	0.073	(0.092)
Age^2	0.036	(0.038)	-0.016	(0.029)
Female	0.007	(0.082)	0.130*	(0.064)
Parent Ethnicity	0.106	(0.132)	0.161	(0.092)
Father's Age	0.011	(0.008)	0.015*	(0.007)
Father's Height	-0.001	(0.003)	0.002	(0.004)
Mother's Age	-0.036**	(0.012)	-0.029**	(0.010)
Mother's Height	0.010	(0.005)	0.017*	(0.007)
Parents' Education—Primary^a^	-0.287*	(0.123)	-0.031	(0.113)
Parents' Education—Secondary^a^	-0.321	(0.191)	-0.063	(0.163)
Household controls				
Household Size	-0.007	(0.021)	0.047*	(0.021)
Household Asset Index	0.144**	(0.046)	0.169***	(0.040)
Rural	0.256	(0.139)	0.138	(0.106)
Geographic Controls				
Southwest and Northwest Region^b^	-0.115	(0.201)	-0.165	(0.196)
Other Region^b^	0.589**	(0.189)	0.523**	(0.194)
Rainfall in 1999	0.000	(0.000)	0.000	(0.000)
Community Cohesion	-0.049	(0.076)	-0.108	(0.069)
Health Care Exclusion	-0.004*	(0.002)	-0.003	(0.001)
Instrumental Variables				
Community Migration Network^c^	-0.018***	(0.002)		
US Destination Wage Rate^d^			0.00002**	(0.000)
Intercept	-2.589**	(0.831)	-5.125***	(1.224)
Wald Chi-Squared(2)^2^	79.33***			

*** *p* ≤ 0.001

** *p* ≤ 0.01

* *p* ≤ 0.05.

^a^ Below primary is the reference category.

^b^ Metropolitan Region is the reference category.

^c^ International migration rate in 2002 times unexpected rainfall in municipality.

^d^ Non-skilled wages in the United States in 1998 times the square of the age of household head.

^1^Standard errors are clustered at the household level. Models are estimated using a probit specification.

^2^Test of joint significance for IVs in both equations.

**Table 3:** Estimated effects of father's migration and receiving remittances on length/height-for-age (HAZ) in Guatemala (N = 3,973).

	Estimate	(SE^1^)
Father migrated internationally	-0.427*	(0.176)
Household received international remittances	0.573	(0.428)
Individual controls		
Age	-1.273***	(0.074)
Age^2	0.296***	(0.023)
Female	0.073	(0.047)
Parent Ethnicity	-0.354***	(0.071)
Father's Age	0.004	(0.004)
Father's Height	0.008	(0.004)
Mother's Age	0.008	(0.006)
Mother's Height	0.028**	(0.009)
Parents' Education—Primary^a^	-0.053	(0.074)
Parents' Education—Secondary^a^	0.139	(0.101)
Household controls		
Household Size	-0.057***	(0.012)
Household Asset Index	0.178***	(0.030)
Rural	-0.122*	(0.063)
Geographic Controls		
Southwest and Northwest Region^b^	0.048	(0.101)
Other Region^b^	-0.202	(0.109)
Rainfall in 1999	0.0002***	(0.000)
Community Cohesion	-0.034	(0.041)
Health Care Exclusion	-0.001	(0.001)
Intercept	-7.221***	(1.777)

*** *p* ≤ 0.001

** *p* ≤ 0.01

* *p* ≤ 0.05.

^a^ Below primary is the reference category.

^b^ Metropolitan Region is the reference category.

^1^Standard errors are clustered at the household level.

Table 3 presents the main results of the analysis. We find that fathers’ international migration is associated with a 0.427 decrease in child HAZ, indicating a greater level of stunting. For the average child residing in a non-migrating, non-remittance receiving household, the 0.427 decrease translates into a 22.1% (-0.427/-1.929) decrease in HAZ. If the father of a child in a non-migrating, remittance-receiving household decides to migrate internationally, the child's HAZ will decrease on average by approximately 27.2% (-0.427/-1.569). In both cases, the child transitions into a stunted state (HAZ ≤ -2). Although the coefficient for the international remittances variable is larger and in the opposite direction, suggesting a positive effect that counterbalances the negative effect of a migrating father, it is not statistically significant at conventional levels.

The results for the control variables align with previous research on the demographic characteristics associated with child health outcomes in Guatemala. We find a quadratic relationship between age and HAZ: HAZ decreases with age, reaches a trough, and then increases thereafter. Mother's height and household wealth are positively associated with HAZ. In contrast, living in a rural area, household size and having a Mayan background are negatively associated with HAZ. To place the importance of fathers’ migration in the context of these background variables, the effect of fathers’ migration on HAZ is just as large as having a Mayan background (-0.354), nearly four times as large as living in a rural area (-0.122), and larger than the effect of moving from the 75th (2.259) to the 25th (0.568) percentile on household wealth ([0.568–2.259] x 0.179 = -0.301). Thus in predicting levels of stunting in Guatemala, a father's migration is equally, if not more significant than the usually cited demographic variables.

## Discussion

For many households in developing countries, migration is an integral part of their livelihood strategy. The concomitant remittances from economic migration have the power to supplement basic household expenditures (food, clothing, medicine) and improve human capital development for many left-behind children. However, migration—especially when fathers leave children behind—can be very disruptive, endangering the provision of sufficient nutrition and lowering health care expenditures, possibly leading to a decline in child well-being. This investigation quantifies at the national level using an IV framework the independent effects of fathers’ migration and remittances on left-behind child growth status in Guatemala.

The key finding in this investigation is the deleterious effect of short-term fathers’ absences due to international migration on a left-behind child’s HAZ growth. Given that the average—nationally representative—Guatemalan child in our sample has a HAZ just above the WHO’s definition of stunting, the potentially harmful effects of fathers’ absences due to economic migration are concerning. The increased likelihood of child undernutrition and its associated long-term repercussions, including poor cognitive development and reduced adult productivity [65], stand in stark contrast to the stated goals of most Guatemalan parents who utilize international economic migration as a means to better the future prospects of their children [66]. For left-behind family members, the loss of a primary breadwinner in addition to borrowing money to finance a trip abroad is likely to pinch food budgets and the ability to grow subsistence food. To compensate, this dynamic may force the left-behind mother to seek gainful employment which indirectly could harm young children through a reduction in child supervision and the possible early reduction/cessation of breastfeeding.

Another compelling finding from this investigation is the lack of significant effects of remittances on HAZ growth. A potential explanation for this result is that international migrant fathers of infant children are likely new migrants and thus must overcome a number of hurdles before they can return meaningful amounts of income to their households. Such obstacles include successfully traveling to the migrant's intended destination, finding stable and gainful employment and avoiding detection by migration authorities in cases where they do not possess legal documents to reside in the destination. Many of these factors can be mitigated to some extent by the presence of strong migration networks connecting a migrant’s community of origin with locations abroad. Social networks can help facilitate the migration journey, such as aiding the migrant with locating a place to live and potential employment opportunities, which reduce the amount of time and expense required to become established in the migrant destination [55, 67, 68]. Despite the beneficial effects of these social networks, positive income flow from migrants to left-behind family members can be hampered by the fact that many economic migrants from Guatemala take out loans to pay the substantial fees demanded by *coyotes* to get them across both the Mexican and US borders. Such loans often require immediate repayment, which substantially reduces the amount that can be returned to migrant-sending families. The average amount of remittances received by the 171 households in our sample that sent a father abroad was $878. In contrast, the average amount of remittances received by households with a child of secondary school age (between 13 and 18), whose internationally migrating fathers are likely to be more established in their migrant destinations, was nearly twice as large ($1,766). While fathers are busily establishing themselves abroad, most households will not have an important laborer that at a minimum could help produce subsistence food. Therefore, left-behind mothers are likely bearing the burden of both agricultural as well as household chores, including caring for children. Considering the lengthy period of time it takes migrants to establish themselves abroad and to send meaningful remittances homeward, we conclude that left-behind households with young children are unlikely to receive sufficient foreign income during the critical three-year period of child development to counteract the harmful effects of fathers’ absences on child growth.

This study does not support Carletto *et al*.’s [24] findings for northwestern Guatemala. They found a negative (beneficial) effect of international migration on stunting in left-behind children. However, their study differs from this one in that they did not separate out the potential harmful effects of parental absences from the benefits of remittances on left-behind children’s nutritional status. A strength of the present study is it shows that when remittances are decoupled from the overall migration effect, fathers’ absences have an overwhelmingly harmful effect on the likelihood of left-behind children being of shortened stature.

A drawback of this investigation is that the ENCOVI data do not provide meaningful migration information beyond the year prior to the survey. Therefore, it is likely that remittances in this study both provide an indication of income flows back to the household and the level of establishment of the migrant at the migration destination. Another data deficiency relates to their cross-sectional nature. Annual panel data that accurately and precisely measure migration events in relation to child births would provide more compelling results. Finally, due to the insufficient sample of migrant mothers, the study cannot speak to the potential effects of a mother's international migration, which arguably may be more harmful to an infant child’s well-being than a father's absence.

Despite these limitations, the study's findings offer several implications as they relate to the strategies that parents in developing countries employ to enhance their children's well-being. In particular, the results from this study show that international economic migration, which is a popular means for improving the livelihood of children in developing countries, may have a permanent negative impact on child well-being under certain conditions. Specifically, we find that a father's international economic migration coinciding with the first three years of a child’s life, which represents the most critical period for physical development, increases the danger of the child becoming stunted. It behooves Guatemalan government and non-governmental organizations interested in migrant health, from both a human welfare as well as a national productivity standpoint, to inform their constituents about the risks of migration on the development of left-behind children. Furthermore, these organizations should urge families with young children to put off the migration of fathers until the three-year development period for all children has been surpassed. And, when possible, they should provide temporary nutritional assistance for migrant households with young children until migrants can successfully establish themselves abroad.

## References

[1] Bierbaum R, Fay M. World development report 2010: development and climate change 2010.

[2] WHO. Global health observatory data repository: country statistics: Guatemala In: Organization WH, editor. 2012.

[3] AdamsRHJr. International remittances and the household: Analysis and review of global evidence. Journal of African Economies. 2006;15:396–425. 10.1093/jafeco/ejl028 .

[4] IOM. Encuesta sobre remesas 2010 ninez y adolescencia Geneva: International Organization for Migration; 2011.

[5] IOM. Encuesta nacional sobre emigración internacional de guatemaltecos Guatemala: OIM 2003:509.

[6] MohapatraS, RathaD, SilwalA. Outlook for Remittance Flows 2011–13: Remittance Flows Recover to pre-Crisis Levels. The World Bank, 2011.

[7] FrankR, WildsmithE. The grass widows of Mexico: Migration and union dissolution in a binational context. Social Forces. 2005;83(3):919–47. 10.1353/sof.2005.0031 .

[8] KanaiaupuniSM, DonatoKM. Migradollars and mortality: The effects of migration on infant survival in Mexico. Demography. 1999;36(3):339–53. 10.2307/2648057 .10472498

[9] HamiltonER, VillarrealA, HummerRA. Mother's, household, and community US migration experience and infant mortality in rural and urban Mexico. Population Research and Policy Review. 2009;28(2):123–42. 10.1007/s11113-008-9097-2 .20047012PMC2677197

[10] McKayD. ‘Sending Dollars Shows Feeling’–Emotions and Economies in Filipino Migration. Mobilities. 2007;2(2):175–94.

[11] SchmeerK. Father absence due to migration and child illness in rural Mexico. Social Science & Medicine. 2009;69(8):1281–6. 10.1016/j.socscimed.2009.07.030 .19699568PMC4070171

[12] de OnisM, OnyangoAW, BorghiE, SiyamA, NishidaC, SiekmannJ. Development of a WHO growth reference for school-aged children and adolescents. Bulletin of the World Health Organization. 2007;85(9):660–7. 1802662110.2471/BLT.07.043497PMC2636412

[13] GrossR, SchoenebergerH, PfeiferH, PreussH. The four dimensions of food and nutrition security: definitions and concepts. SCN News. 2000;20:20–5.

[14] United Nations Children's Fund. Progress for children: A world fit for children: Statistical review: UNICEF; 2007.

[15] HildebrandtN, McKenzieDJ, EsquivelG, SchargrodskyE. The effects of migration on child health in Mexico [with comments]. Economia. 2005:257–89.

[16] NoblesJE. The effects of Mexican migration on sending families: ProQuest; 2007.

[17] PonceJ, OlivieI, OnofaM. The role of international remittances in health outcomes in Ecuador: Prevention and response to shocks. International Migration Review. 2011;45(3):727–45. 10.1111/j.1747-7379.2011.00864.x .22171363

[18] AntónJI. The impact of remittances on nutritional status of children in Ecuador. International Migration Review. 2010;44(2):269–99. 10.1111/j.1747-7379.2010.00806.x .

[19] de BrauwA, MuR. Migration and the overweight and underweight status of children in rural China. Food Policy. 2011;36(1):88–100. 10.1016/j.foodpol.2010.08.001 .

[20] GaoY, LiLP, KimJH, CongdonN, LauJ, GriffithsS. The impact of parental migration on health status and health behaviours among left behind adolescent school children in China. BMC public health. 2010;10(1):56.2012890110.1186/1471-2458-10-56PMC2829003

[21] CarlsonED. The impact of international migration upon the timing of marriage and childbearing. Demography. 1985;22(1):61–72. 3979616

[22] MenjívarC, AgadjanianV. Men's migration and women's lives: Views from rural Armenia and Guatemala*. Social Science Quarterly. 2007;88(5):1243–62.

[23] MartorellR, SchroederDG, RiveraJA, KaplowitzHJ. Patterns of linear growth in rural Guatemalan adolescents and children. Journal of Nutrition. 1995;125(4):S1060–S7. .10.1093/jn/125.suppl_4.1060S7722708

[24] CarlettoC, CovarrubiasK, MaluccioJA. Migration and child growth in rural Guatemala. Food Policy. 2011;36(1):16–27. 10.1016/j.foodpol.2010.08.002 .

[25] StarkO, LucasREB. Migration, remittances, and the family. Economic Development and Cultural Change. 1988;36(3):465–81. 10.1086/451670 .

[26] LucasREB, StarkO. Motivations to remit: Evidence from Botswana. Journal of Political Economy. 1985;93(5):901–18. 10.2307/1833062

[27] VanweyLK. Altruistic and contractual remittances between male and female migrants and households in rural Thailand. Demography. 2004;41(4):739–56. 10.1353/dem.2004.0039 .15622952

[28] BeckerGS, TomesN. Child endowments and quantity and quality of children. Journal of Political Economy. 1976;84(4):S143–S62. 10.1086/260536 .

[29] BeckerGS, LewisHG. Interaction between quantity and quality of children Economics of the family: Marriage, children, and human capital: UMI; 1974 p. 81–90.

[30] DavisJ, Lopez-CarrD. The effects of migrant remittances on population-environment dynamics in migrant origin areas: international migration, fertility, and consumption in highland Guatemala. Population and Environment. 2010;32(2–3):216–37. 10.1007/s11111-010-0128-7 .21258636PMC3003829

[31] GoldsteinS, GoldsteinA. Migration and fertility in peninsular Malaysia: An analysis using life history data: Rand; 1983.

[32] StephenEH, BeanFD. Assimilation, disruption and the fertility of Mexican-origin women in the United States. International Migration Review. 1992;26(1):67–88. 10.2307/2546937 .

[33] StephenL. Zapotec women: Gender, class, and ethnicity in globalized Oaxaca: Duke University Press Books; 2005.

[34] StollD. El Norte or Bust!: How Migration Fever and Microcredit Produced a Financial Crash in a Latin American Town: Rowman & Littlefield Publishers; 2012.

[35] PopkinBM. Time allocation of the mother and child nutrition. Ecology of Food and Nutrition. 1980;9(1):1–13. 10.1080/03670244.1980.9990579 12278625

[36] LevineNE. Womens work and infant feeding—a case from rural Nepal. Ethnology. 1988;27(3):231–51. 10.2307/3773519 .

[37] ToyamaN, WakaiS, NakamuraY, ArifinA. Mother's working status and nutritional status of children under the age of 5 in urban low-income community, Surabaya, Indonesia. Journal of Tropical Pediatrics. 2001;47(3):179–81. 10.1093/tropej/47.3.179 .11419684

[38] LeslieJ. Womens work and child nutrition in the Third-World. World Development. 1988;16(11):1341–62. 10.1016/0305-750x(88)90209-4 .

[39] TuckerK, SanjurD. Maternal employment and child nutrition in Panama. Social Science & Medicine. 1988;26(6):605–12. 10.1016/0277-9536(88)90024-x .3363401

[40] AdlTorre, RushL. The determinants of breastfeeding for Mexican migrant women. International Migration Review. 1987;21(3):728–42. 10.2307/2546619 12314903

[41] WHO. Growth reference 5–19 years 2007 [cited 2011 May 20]. Available from: http://www.who.int/growthref/tools/en/.

[42] WHO. The WHO child growth standards: Macros SPSS 2006 [cited 2011 May 20]. Available from: http://www.who.int/childgrowth/software/en/.

[43] de Onis M. WHO Child Growth Standards: Length/height-for-age, weight-for-age, weight-for-length, weight-for-height and body mass index-for-age: Methods and development. 2006.

[44] Beaton G, Kelly A, Kevany J, Martorell R, Mason J. Appropriate uses of anthropometric indices in children. Nutrition policy discussion paper. 1990.

[45] Marini A, Gragnolati M. Malnutrition and Poverty in Guatemala: World Bank Policy Research Working Paper 2967. Washington DC: World Bank. 2003.

[46] HallmanK, PeraccaS, CatinoJ, RuizM. Multiple disadvantages of Mayan females: the effects of gender, ethnicity, poverty, and residence on education in Guatemala: Population Council; 2006.

[47] Baez J. Does more mean better? Sibling sex composition and the link between family size and children's quality. Available at SSRN 1136273. 2008.

[48] FilmerD, PritchettLH. Estimating wealth effects without expenditure data—Or tears: An application to educational enrollments in states of India. Demography. 2001;38(1):115–32. 10.2307/3088292 .11227840

[49] McKenzieDJ. Measuring inequality with asset indicators. Journal of Population Economics. 2005;18(2):229–60.

[50] McKenzieD, StillmanS, GibsonJ. How Important is Selection? Experimental VS. Non‐Experimental Measures of the Income Gains from Migration. Journal of the European Economic Association. 2010;8(4):913–45.

[51] StillmanS, GibsonJ, McKenzieD. The impact of immigration on child health: experimental evidence from a migration lottery program. Economic Inquiry. 2012;50(1):62–81. 2232904910.1111/j.1465-7295.2009.00284.x

[52] RoodmanD. Estimating fully observed recursive mixed-process models with cmp. Center for Global Development Working Paper. 2009;168:1–57.

[53] CarringtonWJ, DetragiacheE, VishwanathT. Migration with endogenous moving costs. American Economic Review. 1996;86(4):909–30.

[54] TaylorJE, WyattT. The shadow value of migrant remittances, income and inequality in a household‐farm economy. The Journal of Development Studies. 1996;32(6):899–912.

[55] McKenzieD, RapoportH. Network effects and the dynamics of migration and inequality: Theory and evidence from Mexico. Journal of Development Economics. 2007;84(1):1–24. 10.1016/j.jdeveco.2006.11.003 .

[56] YangD, ChoiH. Are remittances insurance? Evidence from rainfall shocks in the Philippines. World Bank Economic Review. 2007;21(2):219–48. 10.1093/wber/lhm003 .

[57] AdamsRH, CuecuechaA. Remittances, household expenditure and investment in Guatemala. World Development. 2010;38(11):1626–41. 10.1016/j.worlddev.2010.03.003 .

[58] MunshiK. Networks in the modern economy: Mexican migrants in the US labor market. The Quarterly Journal of Economics. 2003;118(2):549–99.

[59] Instituto Nacional de Sismología V, Meteorología e Hidrología (INSVMH). http://www.insivumeh.gob.gt/ 2014.

[60] IOM. Encuesta Nacional sobre el Impacto de Remesas Familiares en los Hogares Guatemaltecos. Geneva: International Organization for Migration; 2004.

[61] Bureau of Labor Statistics. Occupational Employment Statistics, accessed on 11/1/2014, http://www.bls.gov/oes/1998/oessrcma.htm. 1998 [11/1/2014]. Available from: http://www.bls.gov/oes/1998/oessrcma.htm.

[62] WoodruffC, ZentenoR. Migration networks and microenterprises in Mexico. Journal of Development Economics. 2007;82(2):509–28.

[63] OsiliUO. Migrants and Housing Investments: Theory and Evidence from Nigeria*. Economic Development and Cultural Change. 2004;52(4):821–49.

[64] BuisML. Stata tip 97: Getting at rho’s and sigma’s. Stata Journal. 2011;11(2):315–7.

[65] MilmanA, FrongilloEA, de OnisM, HwangJY. Differential improvement among countries in child stunting is associated with long-term development and specific interventions. Journal of Nutrition. 2005;135(6):1415–22. .1593044610.1093/jn/135.6.1415

[66] DavisJ. International Migration, Remittances, Fertility, and Development: Quantitative and Qualitative Evidence from Central America: ProQuest; 2010.

[67] McKenzieD, RapoportH. Self-selection patterns in Mexico-US migration: the role of migration networks. The Review of Economics and Statistics. 2010;92(4):811–21.

[68] CurranSR, Rivero-FuentesE. Engendering migrant networks: The case of Mexican migration. Demography. 2003;40(2):289–307. 10.2307/3180802 .12846133

